# The Deep Participation of Zhejiang Private Science and Technology Enterprises in the Integrated Development of the Yangtze River Delta

**DOI:** 10.1155/2022/5667656

**Published:** 2022-04-14

**Authors:** Xiaomin Yin, Siqi Yu

**Affiliations:** ^1^Zhejiang Shuren University, Hangzhou, Zhejiang 310015, China; ^2^College of business administration Zhejiang University of Finance and Economics, Hangzhou, Zhejiang 310018, China

## Abstract

Private science and technology enterprises are the main force in building a high-level innovative province in Zhejiang, and are also the driving force for the province's high-quality integration into the Yangtze River Delta. At present, the integration of private science and technology enterprises in Zhejiang into the Yangtze River Delta has problems such as low integration ratio, high integration difficulty, low integration level, and insufficient integration confidence. The causes of the problem mainly include the concept bottlenecks and capacity limitations of private technology companies, the institutional dilemma of cooperation between regional governments and regional business environment synergy is not high, the role of non-governmental organizations is not fully developed. To create a powerful engine that drives private technology enterprises to deeply participate in the development of the Yangtze River Delta, it should be built and strengthened from the perspective of the main role of enterprises themselves, the role of government guidance, industry associations, and other non-governmental organizations to play the role of service coordination and supervision.

## 1. Introduction

Private science and technology enterprises are private enterprises with a certain number of scientific and technical personnel, independent intellectual property rights, proprietary technologies, or advanced knowledge, mainly engaged in the research, development, production, sales, and service of high-tech and its products. Among them, innovative leading enterprises, high-tech enterprises, science and technology-based small and medium-sized enterprises are the front-runners of private technology enterprises. As of the end of June 2021, Zhejiang province's registered private enterprises were 2,785,400, accounting for 92.5% of the number of enterprises in the province; the province's 22,176 high-tech enterprises in private enterprises accounted for 91.3%, R & D investment accounted for more than 2/3 of the province's enterprise R & D investment. The group of data shows that private technology enterprises have become the main force in building the first province of the national private economy, implementing the first strategy of strengthening the province of innovation and accelerating the construction of a high-level innovative province. At the same time, these enterprises are also a force for life during the “14th Five-Year Plan” period, helping Zhejiang to deeply implement the “Yangtze River Delta Regional Integrated Development Plan Outline” issued by the State Council, to promote the province's high-level integration into the Yangtze River Delta, to create a national digital economy innovation highland, all-round provincial capacity to enhance the development of the Yangtze River Delta world-class city cluster integration of the Golden South Wing of the force for life [1, 2].

Since the integrated development of the Yangtze River Delta region was elevated to a national strategy in 2018, remarkable achievements have been made in the interconnection and interoperability of the Yangtze River Delta transportation, the common construction and sharing of public services, the coordination and mutual promotion of regional planning, and the synergistic protection of the ecological environment, however, the promotion of the strategy is generally still at the “government-led” stage. Private enterprises, especially the most dynamic and growing private science and technology enterprises, have not yet become the real subjects of regional cooperation, and the breadth and depth of such enterprises' participation in integrated development are very limited. At present, as a strong market player supporting most of Zhejiang's science and technology innovation, private science and technology enterprises generally have some problems in the process of participating in the integrated development of the Yangtze River Delta, such as the weak willingness of capital flow across the region, poor free flow of factors, insufficient industrial synergy, and poor performance in R&D cooperation [3].

## 2. Problems in the Process of Integration of Private Technology Enterprises in Zhejiang

At present, under the intertwined influence of the unprecedented changes in a century and the new crown epidemic global pandemic, the world enters a new period of dynamic change, therefore, Zhejiang's economic and social development is facing such problems as increased instability and uncertainty, deep-seated structural contradictions emerge, outstanding supply constraints, and increased downward pressure on the economy [4]. The problems faced by private technology enterprises in the process of improving the level of regional integration and innovation, promoting the full integration of Zhejiang into the Yangtze River Delta, and achieving high-quality integrated development are also intricate and complex. The main points are as follows.

### 2.1. Low Integration Ratio

So far, most of those who have participated in the integrated development of the Yangtze River Delta are the leading backbone enterprises of various industries in the province, and some of them belong to the cultivation targets of the following programs: innovative leading enterprises of Zhejiang Province, national high-tech enterprises (industry innovation-driving ability, possessing core independent intellectual property rights in the industry and belonging to the leading industry enterprises with key support from cities and counties), “Phoenix Action” program version 2.0 (mainly listed enterprises and M&A restructuring enterprises), “Eagle Action” (first-class enterprises with global competitiveness), “Eagle Action” (hidden champion enterprises in subdivided industries). The proportion of ordinary small, medium and micro private technology enterprises that have been and intend to integrate into the development of the Yangtze River Delta is relatively low. According to the research data of this research group, there are 111 private science and technology enterprises operating, investing, and cooperating across regions in the Yangtze River Delta region in the past three years, accounting for 32.74% of the total number of questionnaires (339), and the specific ways of cross-regional development are shown in Table 1. As to the question of whether they intend to make a strategic layout for the integration of Yangtze River Delta in the future, only 11.5% of the enterprises said that they “have a clear plan of action,” 81.42% said “not yet,” and 7.08% said, “Yangtze River Delta integration has nothing to do with enterprise development.” This result shows that the current willingness of enterprises to integrate into the development of the Yangtze River Delta is not high, and the business environment in the Yangtze River Delta region may still be quite different.

### 2.2. High Integration Difficulty

- The Elements Are Difficult to Obtain.
- A tight balance of factors is the objective reality of Zhejiang's long-term economic and social development. Small, medium-sized and micro enterprises account for more than 90% of private enterprises in Zhejiang, and such enterprises have great restrictions on the availability of land required for project investment, financing availability and convenience, scientific and technological innovation ability, market share of leading products or services, industrial chain integration ability, brand integration ability, business recruitment, and intelligence introduction ability, etc. This objectively leads to its difficulty in taking high-quality steps in the integrated development of the Yangtze River Delta [5–7].
- The Phenomenon of Regional Industrial Isomorphism Is Prominent.
- The high similarity coefficient of industrial structure among cities hurts the integration of private technology enterprises into the Yangtze River Delta. We should know that in the process of integrated development, regions with large differences in industrial structure can develop their own characteristic industries to the maximum extent, realize complementary advantages, and promote the circular development of a regional economy. Among the six representative cities in the Yangtze River Delta, Shanghai, Suzhou, Hangzhou, Nanjing, Ningbo, and Hefei have a high degree of similarity in their leading industries, with smart manufacturing, electronic information, biomedicine, new materials, automobiles, and energy chemicals being repeatedly proposed in the industrial plans of each region. Moreover, within some of the same industries, each region sets its development direction on the main part of industrial production with high added value, and less consideration is given to the parts of accessories. There is a lack of specialized division of labor between regions required for efficient industrial integration. As can be seen from Figure 1, the similarity of industrial structure and employment structure within the Yangtze River Delta region is high. In the last decade, although the overall similarity has decreased, it is still not significant.
- The Financing Problem Is Still Prominent.
- In the process of attracting and motivating talents, supporting R&D innovation, implementing transformation and upgrading, and realizing foreign investment, small, medium and micro private technology enterprises in the growth stage all need financial support. At present, bank financing is the most important financing channel for small, medium and micro private technology enterprises in addition to endogenous financing. However, due to the imperfection of the existing laws and regulations and credit guarantee system, many technology enterprises have difficulty in providing collateral that meets the requirements for loans, while the higher risk attributes of technology enterprises themselves make it difficult for them to pass the risk assessment of banks. Therefore, it is very difficult for science and technology enterprises to obtain bank loans [8].
- In addition, from the perspective of the regional financial environment, the financial environment is the short board of Zhejiang's business environment construction. According to the “Yangtze River Delta High-Quality Business Environment Index Report, 2020–2021” prepared and published by Shanghai Hualue Think Tank Group, the indicator item with the biggest gap between Zhejiang and Shanghai is the financial environment. (See Table 2).
- The Policy and Institutional System for Integrated Development are Not Yet Sound.
- The objective existence of local protectionism, market segmentation, and administrative barriers makes it difficult for private technology companies to integrate into the development of the Yangtze River Delta. Enterprises surveyed by the research group generally believe that there are “three hots and three colds” in the current integration process of the Yangtze River Delta, “hot at the top, cold at the grassroots, hot for experts, cold for society, hot for the media, cold for the table.” Strategic planning is a high-rise building, but it is difficult to implement. Some private science and technology enterprises say that this is the inevitable consequence of the government as the main body of the integration model. In this model, local governments may have the mentality of “fertile water does not flow to outsiders' fields” with factors such as talents and capital, or with the motivation of using integrated support policies to obtain more resources for the local area, all localities hope to use the strength of other areas to solve the pain points of local development, but it is difficult to use local resources to solve problems for other areas, resulting in “The local trouble is shared by the region rather than the local advantage.” In the interview, a data technology company in Hangzhou specifically mentioned that data, as the fifth factor of production, is still at the stage of government-led control or even monopoly. Because the Yangtze River Delta region involves three provinces and one city, the data barriers between various places are more, and it is difficult for the data fragments in a silo state to develop into a smooth chain of “data industry” within the Yangtze River Delta region.

### 2.3. The Level of Integration Is Not High

At present, the overall industrial level, added value, and quality and efficiency level of Zhejiang private technology enterprises are not high enough. The problems of broken chains and missing chains in the high-end links of the industrial chain are relatively prominent, and the progress of import substitution is slow, resulting in the integration of enterprises into the development of the Yangtze River Delta industrial level and the modernization of the industrial chain are not high. In addition, Zhejiang private science and technology enterprises' overall R & D investment is insufficient and the gap between the industry R & D investment is obvious. These problems lead to less space for high-quality cooperation between regions through docking high-quality innovation resources in the Yangtze River Delta, building industrial innovation platforms and joint R&D of technologies. It is not fast enough to make use of the leading city Shanghai and the external forces of central cities in the Yangtze River Delta to boost private technology companies to upgrade their industrial levels [9].

### 2.4. Lack of Confidence in the Integration

The current global epidemic situation is intricate and complex, commodity prices are under pressure to rise, and the external environment is unstable and uncertain. In addition to the core industry areas of the digital economy (artificial intelligence, health, strategic emerging, equipment, and high-tech), the profit margins of private technology companies are generally compressed, which makes companies have a high degree of uncertainty and insecurity about future investment. They believe that investment stability in the post-epidemic period is the priority. The investment target within the marginal scope is to choose the low-risk asset allocation method as much as possible, which also reduces the stamina and confidence of entrepreneurs in cross-regional and remote investment to a certain extent.

## 3. Causes of Problems in the Integration Process

The causes of the problem can be analyzed from the perspectives of private technology enterprises themselves, the institutional mechanism of regional intergovernmental cooperation, and the role of non-governmental organizations.

### 3.1. Conceptual Bottlenecks and Capacity Limitations of Private Technology Companies

- Private Technology Enterprises have Cognitive Limitations and Conceptual Bottlenecks.
- At present, many private science and technology enterprises in Zhejiang have limited cognition of the major opportunities of the integrated national strategy and the concept bottleneck of cross-regional cooperation and coordinated development. It is not clear that the integration of the Yangtze River Delta has the dual significance of both opportunities and challenges for enterprises. A considerable number of small, medium and micro private technology companies have a strong “local awareness,” they are highly dependent on regions in their development, lack the awareness and ability to carry out cross-regional long-term strategic layouts, and also lack cross-regional development plans that take the initiative and breakthrough themselves. Therefore, they generally have a fear of the uncertainty of “going out” development [10–12].
- Private Science and Technology Enterprises are Limited by Their Ability to Allocate resources in Different Places.
- The ability to allocate resources in different places mainly depends on the overall organizational management ability of the enterprise. At present, most small and medium-sized private technology enterprises in Zhejiang are still in the transition stage from experience management to scientific management. Although some management systems have been established from scratch, the operation of various specialized functions within the enterprise largely relies on a series of informal behavior control mechanisms. Some private science and technology enterprises follow the traditional family-based and extensive management model, and the scientific utilization of enterprise technology, talents, capital, materials, and other resources is low. In actual work, some private science and technology enterprises are more casual in cost management and capital management, and their quality management standards are not high. Due to the lack of a complete modern enterprise system, it is easy to cause the core resources of the enterprise to be unable to be efficiently allocated or even lead to misallocation of resources. The limitation of resource allocation capacity of private technology enterprises also restricts the space for enterprises to integrate into the development of the Yangtze River Delta to a certain extent.

### 3.2. The Institutional Dilemma of Regional Intergovernmental Cooperation and the Lack of Synergy of the Regional Business Environment

- The Dilemma of a Cooperation System Existing among Regional Governments.
- At present, the relationship between cooperation and competition among various administrative units in the region and the inevitable “paradox of integration” do exist objectively. On the one hand, the three provinces and one city support the national development strategy and actively promote regional integration. They use the hand of the market to promote the continuous blurring and desalination of explicit administrative barriers, attracting more production factors and scarce resources to flow into their respective regions to enhance competitiveness. On the other hand, due to the existence of regional competition, there will be various behaviors that hinder the free flow of production factors, especially the flow of scarce resources to other regions, and form local protectionism, market segmentation, and administrative barriers to varying degrees. For example, in order to hold on to projects and maintain growth, central cities have emerged in an endless stream of subsidy policies, and small and medium-sized cities have continued to promote preferential policies for taxation and land use to win projects and expand their economies. This phenomenon is still common in the Yangtze River Delta region.
- The Synergy of the Business Environment in the Yangtze River Delta Region Is Not High.
- In addition to the different legal environments, the policy environments of the three provinces and one city are also quite different. There are large policy differences between regions in important aspects of the business environment, such as market access, industry standards and norms, industry supervision, safe production, and government procurement. In the Yangtze River Delta region, there are difficulties in policy coordination and convergence to varying degrees, and even policy fights. Taking the enterprise-related special policies that have a direct impact on the vital interests of enterprises as an example, the promulgation of special policies in various places is mostly based on competition and rarely on initiative cooperation now. The claimant is limited to the local administrative region, and the regional inclusive policy is lacking. In addition, the current circulation of resources in the Yangtze River Delta region is not high, and enterprises in the region face many difficulties when relocating and establishing branches, making it difficult to flow efficiently and orderly. In terms of public services, the integrity of public services needs to be improved. At current, the progress of data and information sharing between regions is slow, the number of public affairs matters supporting off-site processing is small and the completion rate is low. Meanwhile, the consistency of the existing business environment evaluation index system also needs to be improved. For example, the scale of administrative law enforcement standards varies across the Yangtze River Delta, and cross-regional comprehensive law enforcement and joint law enforcement are difficult. In a word, although local government services have their highlights and characteristics, they lack an overall system to integrate local standards, and it is difficult to form a unified service specification and work process [13].
- Influence of NGOs Such as Industry Associations
- Industry associations are a consortium of enterprises, with economic and social amphibious properties. They can not only regulate the market, promote economic development, but also unite entrepreneurs and promote industry integration. They are an important force to make up for the lack of government “public order.” However, from the perspective of the requirements of in-depth cooperation in the integration of the Yangtze River Delta, the role of industry associations is faced with problems such as imperfect systems, imperfect operating mechanisms, and too narrow cooperation levels. The work carried out by industry associations still has shortcomings such as “three more and three less”: there are many micro-services, but the macro-level has little drive and guidance for enterprises to integrate into the Yangtze River Delta; there are many liaison activities, but little attention is paid to the problems in the regional coordinated development of enterprises; there are many policy information forwarding, but there is little interpretation and guidance, especially through specific measures to assist enterprises in landing promotion. These all limit the role of industry associations in regional economic integration to a certain extent.

## 4. Countermeasures and Suggestions

To create a powerful engine that drives private technology enterprises to deeply integrate into the Yangtze River Delta, it should be constructed and strengthened from the perspective of three aspects: the main role of the enterprise itself, the guiding role of the government, and the service coordination and supervision role of non-governmental organizations such as industry associations.

### 4.1. Enhancing the Internal Driving Force and Core Competitiveness of Private Technology Enterprises

Zhang Jindong, chairman of Suning Holding Group, believes that “the development of the Yangtze River Delta cannot be separated from the government's planning and guidance, but enterprises are always the main body of development. Therefore, our vast enterprises must take responsibility as soon as possible and become the binder and engine to promote the integrated development of the Yangtze River Delta.” ([How does the Yangtze River Delta unleash scientific and technological innovation? Bank, government, and enterprise tripartite linkage to escort the entire life cycle, https://baijiahao.baidu.com/s?id=1703862866376653325&wfr=spider&for=pc, 2021-06-29.) The inner driving force to stimulate and activate the cross-regional operation and development of private technology enterprises is fundamental to promote the deep participation of enterprises in the integration. The internal driving force is the self-conscious force derived from the internal needs of market entities, and it is the force that plays a decisive role in the development and changes of market entities. How to turn the government's driving force into the internal driving force of the enterprise?.

- Private Science and Technology Enterprises should be deeply aware of the major development opportunities brought by the integrated national strategy to the Yangtze River Delta region and the enterprises themselves.
- The Yangtze River Delta region is rich in scientific and educational resources, has obvious advantages in scientific and technological innovation, and accelerates the promotion of innovative cooperation mechanisms. It brings together nearly 1/3 of the national research and experimental development funds, 1/4 of the “double first-class” construction universities, 1/3 of the major scientific and technological foundations, 1/4 of the national key laboratories, and 1/4 of the national engineering research centers. At the same time, based on the integrated regional advantages, the Yangtze River Delta region is accelerating the formation of several world-class high-tech industrial clusters such as integrated circuits, biomedicine, intelligent manufacturing, and artificial intelligence.
- In the above figure, the blue line represents the dimension of spatial coordination, the red line represents the dimension of innovation output, the gray line represents the dimension of the division of labor and cooperation, and the yellow line represents the dimension of industrial integration. According to Figure 2, since 2018, influenced by the integrated national strategy, the industrial collaboration in the Yangtze River Delta region has entered a stage of rapid development. From the perspective of different dimensions, innovation output has become the main driving force for the coordinated development of the industry. In recent years, the Yangtze River Delta region has taken scientific and technological innovation as the core driving force, strengthened industrial cooperation, integrated industrial chains, and focused on key areas, forming a number of industrial clusters with strong scientific and technological innovation, and attracting more and more private technology enterprises to settle in.
- It should be noted that the competitive advantage of a technology-based enterprise comes from the region and industrial cluster where the enterprise is located. The regional environment is very important for the development of the enterprise. A mature geographical layout, especially the layout of advantageous industrial clusters, can help enterprises connect to the most effective resources at the fastest speed, and endow enterprises with competitive strength in many aspects. To this end, Zhejiang private science and technology enterprises should establish the development concept of openness, mutual benefit, and symbiosis as soon as possible, strengthen the integrated development thinking, seek and act according to the situation, and follow the trend. They should hold the sense of crisis that “missing the integration of the Yangtze River Delta may be missing a rare historic opportunity,” take advantage of the situation to integrate, grasp the opportunities of the Yangtze River Delta, and seize the initiative.
- Private Technology Companies Should Focus on Key Nodes to Enhance Their Core Competitiveness
- In the process of in-depth participation in the regional division of labor and cooperation, private technology enterprises should strengthen strategic thinking, accurately grasp their advantages and positioning, focus on core competitiveness, and deepen key businesses. They also need to stand firm in segmented markets, expand market share, and promote the steady and sustainable development of enterprises. The so-called “cross-border diversification” for short-term interests should be reduced, and efforts should be made to avoid the restriction on long-term investment in enterprise development, which is easily caused by the pursuit of short-term profit maximization.
- The first one is to focus on R&D investment and technological innovation. For private technology companies to deeply integrate into the Yangtze River Delta and achieve leapfrog development, the key is innovation. It should be based on scientific and technological research and development and the transformation and application of achievements, and seize the big market in the Yangtze River Delta with high quality. The second is to forge a long board to supplement the short board to enhance the toughness of the industrial chain and supply chain. They are suggested to grasp the current acceleration of global industrial chain reconstruction and the intelligent upgrading trend of industrial chain, value chain, and supply chain, and to cooperate with the advantageous enterprises in the Yangtze River Delta to improve the scale and energy level of the industrial chain. With the help of the economic aggregate and radiation potential of the Yangtze River Delta, it is more promising to build a more resilient industrial chain and supply chain system in the process of regional integration and development. The third is to focus on brand strategy and take the road of high-quality brand development. The brand economy is becoming an important force to accelerate the integration of the Yangtze River Delta and an important node of the enterprise integration strategy. Private technology enterprises should strengthen the integrated development path of scientific and technological innovation, trademark application, and brand promotion. Specifically, they should achieve corporate brands with independent innovation, shape corporate brands with the spirit of craftsmen, accelerate the transformation of innovation achievements into independent trademark brands, and carry out brand cooperation in the Yangtze River Delta region around the cross-border mutual promotion of brands, direct product procurement, and brand implantation. The fourth is to accelerate the establishment of a modern enterprise system in regional cooperation and linkage. Private science and technology enterprises should improve and perfect a modern corporate governance system with the board of directors, management, and board of supervisors as the backbone around the principles of scientific decision-making, quick response, smooth operation, efficient execution, and controllable costs. In addition, it is equally important to continuously optimize the organizational structure adjustment mechanism, business transformation and operation mechanism, and the intergenerational inheritance mechanism of family businesses.

### 4.2. Forming a Joint Force to Promote the Participation of Private Science and Technology Enterprises through the Government's Guiding Service Guarantee Role

- The Construction of a Market-Led Cooperation Mechanism in the Yangtze River Delta Region is the Foundation.
- Only on this mechanism can the integration process of the Yangtze River Delta be more efficient and transparent. “Compared with the regional attributes of the government, the power of the market is naturally integrated. Therefore, to return to the essence of integration, it is necessary to give more play to the role of the market. At the government level, the focus should be on the co-construction and sharing of public facilities, the creation of public platforms, and unification of market rules, standards, and supervision.” (Li Ying: “Some Reflections on the Integration of Adjacent Areas in Metropolitan Areas,” https://www.sohu.com/a/481631815_121106832, 2021-08-05.) Adequate market competition is the micro-mechanism for the formation of the integrated development of the Yangtze River Delta region. The promotion of high-quality integration in the Yangtze River Delta should be mainly based on market factors. It is necessary to continuously overcome and eliminate institutional obstacles that affect the free flow of resources and factors, to finally achieve market opening, full market competition, and market-determined resource allocation. A mechanism of self-association, self-coordination, and self-development of market entities between regions should be established, and the endogenous effect of promoting regional economic integration should be simultaneously generated in the cross-regional development of market entities. Of course, the government should adhere to the combination of decentralization and integration, regulate competition while liberalizing the market, and coordinate the process of regional integration in the Yangtze River Delta by building unified competition rules.
- It Is an Inevitable Requirement to Strive to Break through the Administrative Barriers between Regions.
- To promote the integration of the Yangtze River Delta, efforts must be made to break through administrative barriers. Governments across the Yangtze River Delta should take a broad view of society and the attitude of “open-minded, wise, and modest” as required by modern governments to look at the overall situation and seek out the general situation, and work together as a group towards the goal of the top-level design of the central decision-making. The concept of a win-win regional government “community” guides the creation of an open governance system in the Yangtze River Delta. The first is to promote the coordinated governance of governments across the Yangtze River Delta. Coordinated government governance is an important manifestation of the integration of the Yangtze River Delta in the main dimension, and it is also an effective means to break through the administrative barriers between regions. To realize the coordinated governance under the premise of “not breaking administrative subordination and breaking administrative boundaries” in the Yangtze River Delta region, the overall guidance and comprehensive coordination of the “Leading Group for Promoting the Integrated Development of the Yangtze River Delta” and the “Yangtze River Delta Regional Cooperation Office” should be fully utilized at present. With the direction of breaking through administrative barriers and promoting the integration of factor markets, the government can study and introduce supporting policies and comprehensive reform measures in the Yangtze River Delta in terms of innovation, industry, talent, investment, and finance. The second is to further relax investment access restrictions for private technology enterprises in the Yangtze River Delta region. Local governments should follow the spirit of the “Opinions of the Central Committee of the Communist Party of China and the State Council on Creating a Better Development Environment to Support the Reform and Development of Private Enterprises” and the “Implementation Opinions on Supporting Private Enterprises to Accelerate Reform, Development, Transformation and Upgrading” issued by six departments including the National Development and Reform Commission and the Ministry of Science and Technology, fully implement the policies and measures to relax the market access of private enterprises in the Yangtze River Delta region. To be specific, local governments ought to streamline the administrative approval items for market access, continue to track and regularly evaluate the implementation of relevant market access policies, and comprehensively investigate and systematically clear all kinds of explicit and implicit barriers. The third is to establish and improve the regional interest coordination mechanism that is the key to breaking through the administrative barriers in the Yangtze River Delta. As the highest representative of regional interests, the government should actively explore and establish interest coordination mechanisms such as communication and negotiation with other local governments in the region while avoiding excessive involvement in the microeconomic field as much as possible. Efforts should be made to expand cooperation fields, enrich cooperation paths, and innovate cooperation forms. To solve the problem of “1 + 1+1 + 1 > 4” as a guide, the government should also actively explore the fiscal and tax sharing mechanism between regions in the Yangtze River Delta region, and the cost-sharing mechanism for high-quality public services.
- It Is of Profound Significance to Improve the Compatibility of the Business Environment in the Yangtze River Delta Region.
- All regions in the Yangtze River Delta should think about the overall optimization of the regional business environment from a broader perspective and dimension. They can use the Yangtze River Delta Integrated Development Demonstration Zone as a “model room” to explore the further unification of the Yangtze River Delta region in terms of market, resources, and policy systems, and the in-depth integration of the main sectors of the business environment such as market environment, government services, law enforcement, and legal protection. It is suggested that the three provinces and one city can benchmark the business environment evaluation index system of the World Bank and the National Development and Reform Commission, and take the lead in exploring the establishment of a regional business environment evaluation index system in the Yangtze River Delta based on the actual situation of the Yangtze River Delta region.
- The Government Should Encourage Cross-Regional Mergers and Acquisitions of Private Technology Companies.
- The merger and reorganization of regional enterprises is the most effective micro-mechanism in the development of economic integration, it is also an important factor for enabling technology enterprises to achieve high-quality and efficient development with the help of the capital market and leading more social capital to invest in innovative industries to enhance Zhejiang's overall technological competitiveness. Therefore, the Zhejiang government departments should increase efforts to guide and encourage private technology enterprises to implement cross-regional mergers and acquisitions in the capital market, especially to support high-tech private enterprises to achieve “capital, technology, industry” linkage through mergers and acquisitions. Mergers and acquisitions should be taken as an important tool to actively promote the accelerated integration of private technology enterprises into the integrated development process of the Yangtze River Delta and reshape the regional market, and give full play to the structural effect, competition coordination effect, and self-cleaning effect of the market.
- The Cluster Development of Private Technology Enterprises in the Yangtze River Delta Should Be Supported.
- Local governments should actively guide private technology enterprises in Zhejiang to focus on the advantages of digital economic development, formulate the future industry promotion plan in the Yangtze River Delta. Technological research in areas such as brain-like chips, artificial intelligence, quantum information, future networks, and intelligent perception should be further strengthened, and the construction of digital economic industrial clusters such as visual intelligence, cloud computing, big data, and e-commerce should also be accelerated. In addition, it is necessary to further implement the Zhejiang Yangtze River Delta industrial chain supplementing and strengthening action, sort out the industrial chain map, analyze the risk points of chain breakage, and propose measures for supplementing, solidifying, and strengthening the chain. For private technology enterprises with significant upstream and downstream leading roles and supply chain integration capabilities, it is necessary to implement the “chain master” enterprise cultivation plan as soon as possible. Different policies shall be given to the existing “chain master” enterprises, the “chain master” enterprises under construction, and the recruited “chain master” enterprises. Finally, by focusing on the leading projects, the main projects of the industrial chain, and the strategic emerging industry projects in the Yangtze River Delta region, the scale situation of attracting one, bringing a group, and forming a cluster will be formed.
- It Is Very Important to Improve the Financial Credit Support System for Private Technology Enterprises to Integrate into the Yangtze River Delta.
- Financial institutions should actively explore the integration plan of financial services in the Yangtze River Delta, speed up the construction of an industrial financial cluster business model, accelerate digital operations. Meanwhile, they ought to increase the credit extension of small, medium and micro private technology enterprises in the Yangtze River Delta and improve the customer experience of private banks in the Yangtze River Delta, to fully help private technology enterprises to deeply integrate into the Yangtze River Delta. Financial institutions can also customize exclusive financial support programs for technology-based private enterprises, and design unique and differentiated products such as “Equipment Access,” “Technology Express Loans,” and “Cross-border M&A” direct loans for them.

### 4.3. The Role of Industry Associations and Other NGOs in Service Coordination and Supervision

The integrated development of the Yangtze River Delta region requires not only the top-down promotion of the government but also the bottom-up support from the market and society. For non-governmental organizations such as industry associations, it is necessary to rethink and reposition their functions in promoting the integrated development of the Yangtze River Delta region and play an active role by their professional advantages and civil representation. The roles of NGOs in the integrated development of the Yangtze River Delta region are as follows:

The first is to play the role of the industry service function, including promoting the regional industrial transfer and optimizing industrial layout; building a common technology and service platform for the Yangtze River Delta industry and establishing a regional innovation alliance; promoting the exchange and flow of talents in the Yangtze River Delta. The second is to play the role of industry representative, including promoting the optimization of industrial policies in the Yangtze River Delta; strengthening negotiations and cooperation with upstream and downstream industries, and establishing regional cross-industry alliances. By giving full play to the industry representative function, industry associations can lead and drive enterprises to integrate into the development of the Yangtze River Delta as soon as possible. The third is to play the role of industry coordination, including promoting communication and coordination inside and outside the industry in the Yangtze River Delta, following up on difficult issues in the coordinated development of enterprises in the region, and resolving various conflicts and disputes. The fourth is to give full play to the self-discipline function of the industry, including establishing an industry convention in the Yangtze River Delta, developing the integrity of industry enterprises, formulating regional industry standards, protecting intellectual property rights, and assisting the government in industry supervision. Through the construction of relevant standards, there are specific measures in various industries that can guide the implementation of enterprises.

## Figures and Tables

**Figure 1:** Similarity of industrial structure and employment structure in the Yangtze River Delta.

**Figure 2:** The innovation and integration of industries in the Yangtze River Delta has entered an accelerated period (unit: point).

**Table 1:** What are the main cross-regional operation/investment/cooperation methods of your company in the past three years? [Multiple Choice Questions].

Option	Subtotal	Proportion (%)
Cooperation in scientific and technological innovation and transfer and transformation of patent projects	51	46.43
Participating in the construction of “enclave”	8	7.14
Establishing subsidiaries	20	17.86
Business outsourcing	16	14.29
Shareholding, holding, or wholly-owned acquisition	16	14.29
Others	36	32.14
The number of private technology entrepreneurs who effectively filled in this question	111	

*Note.* This question requires private technology companies with experience in cooperation in the Yangtze River Delta region to fill in, and the number of validly filled companies is 111 (the total number of questionnaires for the project is 339).

**Table 2:** The secondary index scores of the Yangtze River Delta high-quality business environment index and the gap between Zhejiang and the three places.

Indicators	Public service		Innovation environment		Human environment		Market environment		Financial environment	
	Infrastructure	Government affairs environment	Institutional investment	Regional innovation	Human level	Talent service	Market potential	Economic activity	Financial development	Financial support
Zhejiang	72.5	87.5	85.5	68.0	70.0	70.0	69.0	69.0	68.5	65.0
Shanghai	100.0	90.0	67.5	100.0	100.0	100.0	79.0	97.5	85.0	100.0
Jiangsu	74.8	77.2	78.0	68.0	70.0	72.0	68.4	78.4	71.2	62.8
Anhui	70.5	82.5	77.5	69.0	64.0	65.0	69.5	70.0	66.0	60.5
Zhejiang-Shanghai	−27.5	−2.5	18.0	−32.0	−30.0	−30.0	−10.0	−28.5	−16.5	−35.0
Zhejiang- Jiangsu	−2.3	10.3	7.5	0.0	0.0	−2.0	0.6	−9.4	−2.7	2.2
Zhejiang- Anhui	2.0	5.0	8.0	−1.0	6.0	5.0	−0.5	−1.0	2.5	4.5

Source: Shanghai Hualue Think Tank Group: 2020–2021 “Yangtze River Delta High-Quality Business Environment Index Report,” released on December 18, 2020.

## Data Availability

The data used to support the findings of this study are available from the corresponding author upon request.
